The article "Vitamin C in Health and Disease: Its Role in the Metabolism of Cells and Redox State in the Brain" was published in 2015. Journal: Front Physiol.

# Vitamin C in Health and Disease: Its Role in the Metabolism of Cells and Redox State in the Brain

**DOI:** 10.3389/fphys.2015.00397

**Published:** 2015-12-23

**Authors:** Rodrigo Figueroa-Méndez, Selva Rivas-Arancibia

**Affiliations:** Laboratorio de Estrés Oxidativo y Plasticidad Cerebral, Departamento de Fisiología, Facultad de Medicina, Universidad Nacional Autónoma de MéxicoMéxico, Mexico

**Keywords:** vitamin C, pharmacokinetics, neurophysiology, oxidative stress, learning and memory processes

## Abstract

Ever since Linus Pauling published his studies, the effects of vitamin C have been surrounded by contradictory results. This may be because its effects depend on a number of factors such as the redox state of the body, the dose used, and also on the tissue metabolism. This review deals with vitamin C pharmacokinetics and its participation in neurophysiological processes, as well as its role in the maintenance of redox balance. The distribution and the concentration of vitamin C in the organs depend on the ascorbate requirements of each and on the tissue distribution of sodium-dependent vitamin C transporter 1 and 2 (SVCT1 and SVCT2). This determines the specific distribution pattern of vitamin C in the body. Vitamin C is involved in the physiology of the nervous system, including the support and the structure of the neurons, the processes of differentiation, maturation, and neuronal survival; the synthesis of catecholamine, and the modulation of neurotransmission. This antioxidant interacts with self-recycling mechanisms, including its participation in the endogenous antioxidant system. We conclude that the pharmacokinetic properties of ascorbate are related to the redox state and its functions and effects in tissues.

## Introduction

Vitamin C is involved in the maintenance of body functions. However, there is a great deal of studies that show contradictory results about its effects. From the time it was first isolated in 1928, numerous studies have been done on its biochemical and pharmacokinetic properties, its functions and even the role of this molecule in neurophysiology. It is important to identify the role vitamin C has in the maintenance of oxide/reduction (redox) balance, as well as the possible effect it may have on the treatment of chronic degenerative diseases, autoimmune diseases and cancer. The purpose of this review is to update the current state of knowledge on vitamin C and the relevance it has in medicine since its effects are yet to be fully understood.

### Ascorbic acid, ascorbate, and vitamin C

Ascorbic acid is a neutrally charged molecule which can be protonated and become ascorbate. Depending on the pH of the medium in which it is located, ascorbic acid may lose the hydrogen ions attached to one of its two ionizable groups located at carbons 2′ and 3′, generating ascorbate monoanion or dianion (Tolbert et al., 1975; Markarian and Sargsyan, 2011; Du et al., 2012; Figure 1). Ascorbic acid is a white crystalline solid soluble in water; one of its important roles lies in its biochemical function in redox processes. When we talk of vitamin C, we refer to the group of ascorbic acid analogs that can be both synthetic and natural molecules (Huh et al., 1998; Raić-Mlić et al., 2000; Yamamoto et al., 2002).

**Figure 1:** **pH-dependent forms of vitamin C**. At pH 7, close to plasma pH, the predominant form of vitamin C will be ascorbate monoanion, followed by ascorbic acid and, in very low concentrations, ascorbate dianion (0.005%); in an acidic pH, the predominant form will be ascorbic acid.

### Biosynthesis

Plants and many animals have the capacity to synthesize ascorbic acid through several biosynthesis pathways (Figure 2). In fish, amphibians, reptiles, and bird species belonging to older taxonomic orders the enzymes involved in vitamin C biosynthesis are located mainly in the kidneys, while in mammals and bird species from more recent orders these enzymes are found mainly in the liver (Grollman and Lehninger, 1957; Chatterjee et al., 1961). However, species such as teleost fish, some passeriform birds, guinea pigs, and some primates like humans, have lost the ability to synthesize ascorbic acid (Grollman and Lehninger, 1957; Linster and Van Schaftingen, 2007). The enzyme responsible for this deficiency is L-gulonolactone oxidase, which is highly mutated in humans despite having the gene encoding the protein, referred to as a pseudogene (Nishikimi and Yagi, 1991; Nishikimi et al., 1994; Valpuesta and Botella, 2004). For this reason, these species require ascorbic acid from the diet, mainly that synthesized by plants (Figure 2).

**Figure 2:** **Vitamin C biosynthesis**. The initial metabolite of both pathways is glucose, which through a sequence of reactions involving an energy expenditure by the cell, synthesizes L-ascorbic acid. 1, Glucose-6-phosphate isomerase; 2, Mannose-6-phosphate isomerase; 3, Phosphomannomutase; 4, GDPD-mannose pyrophosphorylase; 5, GDP-D-mannose-3,5-epimerase; 6, Phosphodiesterase; 7, Sugar phosphatase; 8, L-galactose dehydrogenase; 1′, Phosphoglucomutase; 2′, UDP-glucose pyrophosphorylase; 3′, UDP-glucose dehydrogenase; 4′, Glucuronate-1-phosphate uridylyltransferase and Glucurono kinase; 5′, Glucuronate reductase; 6′, Aldono-lactonase.

## Pharmacokinetics

### Absorption mechanisms

Ascorbate is the main form of vitamin C in the human body (Rumsey and Levine, 1998). This molecule acts as a co-substrate for several enzymes that are important for the functioning of the organism. Its activity as an antioxidant includes the ability to be reversibly oxidized to ascorbyl radical and then to dehydroascorbate (DHA; Wells and Xu, 1994).

Both forms are ingested in the diet, since ascorbate can be oxidized in the gastrointestinal tract (GIT) by the presence of other substances that act as oxidizing agents [e.g., Iron (F3+) and some flavonoids] (Wilson, 2002). Ascorbate may also be oxidized as a result of food processing, either by cooking techniques or by improper storage techniques in the case of packaged products (Wilson, 2002).

### Sodium-dependent vitamin C transporters (SVCTs)

Two sodium-dependent vitamin C transporters have been described, SVCT1 and SVCT2; both are glycoproteins that transport ascorbate into the cell. SVCT1 is encoded by a gene that belongs to the family of solute carriers, group 23A, member 1 (SLC23A1) of 1797 bp, while the SLC23A2 gene of 1952 bp encodes SVCT2 (Daruwala et al., 1999). In addition, it has been documented that SVCT1 transports ascorbate nine times faster (Steiling et al., 2007) than SVCT2, while the latter has a higher affinity for ascorbate, with an apparent Km of 21.3 uM for SVCT2 and of 252.0 uM for SVCT1 (Daruwala et al., 1999; Figure 3).

**Figure 3:** **Influx and efflux mechanisms. (3.1)** The type of SVCT transporter depends on the characteristics and requirements in each cell, SVCT2 being more frequent in tissues that require a constant supply of ascorbate, even under vitamin C deficiency conditions, while SVCT1 is more frequent in cells responsible for tissue distribution of ascorbate. **(3.2)** Ascorbate transportation into the enterocyte occurs through SVCT1, coupled to a Na+/K+ATPase. **(3.3)** Under conditions of restricted ascorbic acid intake, the supply of ascorbate to the cell is carried out through the SVCT2 located in the basolateral membrane, which is also coupled to a Na+/K+ATPase. **(3.4)** DHA is transported into the enterocyte via GLUT transporters. **(3.5)** Within the enterocyte, DHA is reduced to ascorbate, then exits the cell and spreads to the capillaries through the extracellular space.

The properties of these two transporters are likely to be the explanation of their tissue distribution. SVCT1 is found mostly in epithelial tissues (e.g., small intestine and proximal tubule of the nephron), where the transport of ascorbate is greater than that required by the cells. On the other hand, SVCT2 is found mainly in brain, skeletal muscle, placenta, and eye, where the contribution of ascorbate is tightly controlled to maintain adequate tissue concentrations (Wilson, 2005; Figure 3.1). The transport mediated by these glycoproteins is a secondary active, saturable Na+-dependent transport (Tsukaguchi et al., 1999).

### Glucose transporters (GLUTs)

There have been described 14 GLUT proteins belonging to the family of solute carriers, group 2A (SLC2A; Mueckler and Thorens, 2013). Within this group, only GLUT1 and GLUT3, and to a lesser extent GLUT4, have been found to have the capacity to transport DHA (Li and Schellhorn, 2007). However, the ability of GLUT8 and GLUT2 to transport DHA into rat enterocytes has been shown (Corpe et al., 2013); this is important because GLUT8 and GLUT2 are also present in the human small intestine (Doege et al., 2000; Mueckler and Thorens, 2013).

Each of these transporters has its own characteristics and a specific tissue distribution. The GLUT1 isoform is widely expressed in the body; its presence in endothelial cells of the blood-brain barrier may contribute to the maintenance of concentration of ascorbate in the brain (Li and Schellhorn, 2007). GLUT3 is a high affinity transporter (low Km) that initially was thought to be only present in neuronal cells, but now has been found in sperm, embryos, and leukocytes (Mueckler, 1994; Simpson et al., 2008). GLUT4 is expressed mainly in adipocytes and in skeletal and cardiac muscles; an important feature of this transporter is that it is found mostly within intracellular vesicles which attach to the plasma membrane in response to insulin (Mueckler, 1994). GLUT 2 has the peculiarity of being a low affinity transporter (Km ~ 17 mM); it is found in hepatocytes, enterocytes of the small intestine, proximal tubular cells, and β-pancreatic cells (Mueckler, 1994). GLUT8 is found in skeletal muscle, heart, small intestine, brain, and testis; its expression in testis can be suppressed by estrogens (Doege et al., 2000) Therefore, DHA transport is performed by a facilitated, saturable diffusion mechanism mediated by some GLUT transporters, which, unlike the transport of ascorbate, is Na+ independent.

### Mechanisms of entry into enterocytes

Both ascorbate and DHA can enter enterocytes via SVCT and GLUT transporters, respectively. The absorption pattern of ascorbate is opposite to that of glucose as ascorbate is better absorbed in the most distal segments (ileum) of the small intestine and, in smaller quantities, in the most proximal segments (duodenum). For its part, DHA is better absorbed in the jejunum while very little is absorbed in the distal segments of the ileum (Malo and Wilson, 2000).

One study showed that both SVCT1 and SVCT2 are expressed by enterocytes, but their distribution in the plasma membrane is polarized, as SVCT1 is found in the apical side of cells (Figure 3.2) and SVCT2 is present in the basolateral membrane (Boyer et al., 2005; Figure 3.3).

Part of the DHA absorbed corresponds to ascorbate oxidized in the lumen of the gastrointestinal tract (Wilson, 2002; Figure 3.4). It is yet to be defined which GLUT transporters are responsible for transporting DHA into the enterocyte. Although Corpe et al. proposed that GLUT2 and GLUT8 might be the transporters (Corpe et al., 2013), their study was performed using rats; additionally, other studies hold contradictory views. Some even point out that GLUT2 is not a DHA transporter (Cura and Carruthers, 2012), but others show that it is (Mardones et al., 2011).

### Efflux mechanisms

Although some hypotheses have been proposed, it is still unknown how ascorbate exits the cells. One of the hypotheses holds that epithelial enterocytes and renal proximal tubule cells swell when transporting some metabolites (Wilson, 2002, 2005). This process could activate volume sensitive anion channels (VSAC) located in the basolateral membrane which would allow the exit of ascorbate from inside the cell. It must be said that even though the effect has been observed, the protein has not been identified in enterocytes yet (Wilson, 2002, 2005; Corti et al., 2010; Figure 3.5). The VSAC are a family of membrane proteins that mediate the passive transport of organic anions in response to changes in intracellular osmolarity (Jackson and Strange, 1993; Strange and Jackson, 1995). This mechanism has been demonstrated in cultured astrocytes (Siushansian et al., 1996) and it is very likely to be present in enterocytes as well.

Another mechanism that has been proposed as transporter is an ascorbate-glutamate hetero-exchange (Grûnewald and Fillenz, 1984); however, some researchers believe its existence is unlikely and attribute the glutamate effect to the fact that glutamate favors the entry of Na+/Cl- activating N-methyl-D-aspartate (NMDA) and non-NMDA receptors, glutamate transporters and voltage-gated sodium channels (Vogler et al., 2013), causing the cell to swell and to activate VSAC (Corti et al., 2010). Ascorbate release, mediated by an exocytosis process (Von Zastrow et al., 1984) or by its passage through gap junctions (Wilson, 2005) has also been proposed as transporter. As for DHA, it is reduced to ascorbate inside the enterocyte by complex recycling mechanisms; then it exits the cell and goes into the extracellular space where it reaches the bloodstream through fenestrated capillaries that supply the mucosa of the small intestine (Wilson, 2002, 2005).

### Tissue distribution

The organs with the highest concentration of ascorbate are the adrenal glands (550 mg/kg), the brain (140 mg/kg), the liver (125 mg/kg), and in terms of size, the skeletal muscle with a concentration of 35 mg/kg (Richelle et al., 2006). The function performed by ascorbate in each cell of these organs will determine the type of transporter that is best suited for their local requirements. Regarding the central nervous system (CNS), the ascorbate located in the cerebrospinal fluid diffuses freely into the extracellular space of neurons and glia, where it is captured by both cell types via SVCT2 (except for astrocytes; García Mde et al., 2005; Savini et al., 2008; Gess et al., 2010). SVCT2 is the main transporter in the adrenal glands, (Savini et al., 2008); it maintains high concentrations of ascorbate in the chromaffin cells of the adrenal medulla, which are essential for the synthesis of catecholamines. SVCT1 is the most abundant transporter in the liver although SVCT2 is also expressed. A study carried out by Michels, Joisher and Hagen showed a decrease in the ascorbate uptake in rat hepatocytes due to a lower expression of the mRNA of SVCT1 associated with age (Michels et al., 2003).

In order for ascorbate to be able to reach tissues, it must go through the endothelial barrier of each tissue. One report demonstrated that ascorbate transport takes place primarily through a paracellular pathway (except in CNS) since transcellular transport is not correlated with the ascorbate transferred across the endothelium. Thus, ascorbate transport will depend on the narrowness of the space that exists between endothelial cells. This suggests that the process may be influenced by the rigidity conferred by ascorbate to the cytoskeleton of the cells forming the barrier (May et al., 2009).

## Vitamin C and CNS

Ascorbate functions in the nervous system can be divided as follows: firstly, the interaction of ascorbate with the blood-brain barrier as well as its medical implications; secondly, its effects on the process of neuronal differentiation, maturation and survival; thirdly, its effect on modulating neurotransmission and its participation in catecholamine synthesis. Finally, it has an antioxidant effect and it also plays a role in the learning and memory process as well as in the structure and support of the nervous system.

### Blood-brain barrier

The blood-brain barrier is formed by three cells: the endothelium of the microvasculature of the brain, pericytes, and astrocytes. It has been proposed that astrocytes may induce the formation of the tight junctions between endothelial cells and influence the characteristic phenotype of the transporters of the blood-brain barrier (e.g., GLUT1 and amino acid transporter L1; Abbott, 2002). For their part, pericytes appear to be involved in both maintaining the structural integrity of the vessel wall and regulating angiogenesis; they also seem to have a neuroimmunological effect due to their ability to phagocytize (Ballabh et al., 2004).

The main function of the blood-brain barrier is to maintain the internal microenvironment of the CNS, mediating the selective transport of nutrients, ions, waste products, drugs, and other substances (Abbott et al., 2006). Although ascorbate can penetrate into the CNS through the choroid plexus, it cannot cross through the blood-brain barrier because the tight junctions of the endothelium do not allow ascorbate transport through the paracellular pathway (Harrison and May, 2009). What is more, SVCT2 is not expressed in these cells (Qiao and May, 2009). Even though DHA can cross the blood-brain barrier through GLUT1 (Agus et al., 1997), it is not the main pathway through which ascorbate reaches the CNS; nevertheless it could be an important route from a therapeutic point of view. Huang et al. administered different doses of DHA intravenously before and after the induction of a stroke in mice. They found that DHA had a neuroprotective effect directly proportional to the dose administered. The protective effect was significant whether DHA was injected before or after the stroke (Huang et al., 2001).

Ascorbate distribution in the brain is not uniform. The amygdala, the hippocampus and the hypothalamus are the brain regions with the highest concentration of vitamin C, but even in these structures the distribution is not homogeneous (Mefford et al., 1981). For example, the medial nucleus has a greater concentration of ascorbate in the hypothalamus than in either the preoptic nucleus or the posterior nucleus (Mefford et al., 1981). The *substantia nigra* is the brain region with the lowest concentration of ascorbate (Grümewald, 1993), which could be considered a susceptibility factor for oxidative stress if we consider that the synthesis of dopamine is pro-oxidant and needs ascorbate. Therefore, the requirements of ascorbate that dopaminergic neurons need may be the cause of the low ascorbate levels found in this brain structure.

### Vitamin C and neuronal differentiation, maturation, and survival

The effect of ascorbate on the differentiation of embryonic stem cells into neurons *in vitro* is associated with an increase in the expression of genes involved in this process (Harrison and May, 2009). Lee et al. found that cells treated with ascorbate significantly increased the expression of NeuroD, Notch, BMP2, and BMP7, genes associated with the differentiation of neuronal and astrocytic cells. The same study demonstrated that vitamin E and glutathione do not have the same effect as ascorbate on neuronal cell differentiation so that the mechanism involved might not be directly related with its antioxidant effect (Lee et al., 2003). An increase in neurite formation in neurons *in vitro* due to the potentiating effect of 2-glucoside-L-ascorbic acid (ascorbate analog) on the nerve growth factor (NGF) has also been shown. This is an effect that the authors also attributed to a different mechanism given its antioxidant properties (Haramoto et al., 2008). An increase in the expression of brain-derived neurotrophic factor (BDNF) associated to the presence of ascorbate has also been observed in cell culture. BDNF activates the Ras-MAP kinase pathway, which contributes to cell survival by enhancing the expression of the enzymes of the endogenous antioxidant system [superoxide dismutase (SOD), glutathione peroxidase and glutathione reductase] (Grant et al., 2005).

### Vitamin C, catecholamine biosynthesis and modulation of neurotransmission

As it was said before, ascorbate plays an important role in the synthesis of catecholamines, particularly dopamine and norepinephrine. Seitz et al. proposed that the modulatory effect of ascorbate can be divided into short and a long term. The short term refers to its participation as a co-substrate for tyrosine hydroxylase and dopamine-β-hydroxylase; and the long term effect, to the increased gene expression of tyrosine hydroxylase, probably through a mechanism that involves an increase in intracellular cAMP; however, the latter is still just a hypothesis (Seitz et al., 1998). Studies in ascorbate-deficient guinea pigs showed that the subjects had high dopamine and low norepinephrine levels due to alterations in the catalysis mediated by dopamine-β-hydroxylase; the levels were normalized even with low ascorbate concentration in the brain (Harrison and May, 2009). There are also reports which state that ascorbate promotes and maintains the differentiation of dopaminergic cells derived from midbrain neural precursors *in vitro* (Yan et al., 2001). Yu et al. carried out a study to identify the genes involved in the differentiation of these cells, and they found the upregulation of up to 92 genes and the downregulation of 118 genes, varying according to the stage of cell differentiation (Yu et al., 2004). An increase in the susceptibility to excitotoxicity mediated by the NMDA glutamate receptor in mice with SVCT2 deficiency has also been shown (Qiu et al., 2007). This mechanism can be explained either by an antioxidant effect of ascorbate on reactive oxygen species (ROS) generated by the activation of the receptor or by the interaction of ascorbate with a redox modulation site at the NMDA receptor level (Majewska et al., 1990). Other authors have described the effect of ascorbate as an inductor of the liberation of gonadotropins (luteinizing hormone and follicle-stimulating hormone) (Karanth et al., 2001). What they propose is that ascorbate released by the vesicles of the gonadotrope cells is recaptured by SVCT2 via an unknown mechanism and facilitates the entry of Ca^2+^ into the cell, which interacts with calmodulin and induces an increase in the activity of neuronal nitric oxide synthase (nNOS). Nitric oxide (NO) activates guanylate cyclase increasing the amount of cGMP. Finally, cGMP activates the protein kinase C (PKC), leading to exocytosis of gonadotropine (Karanth et al., 2001).

### Vitamin C, learning, and memory

Parle and Dhingra injected doses of 60 and 120 mg/kg of ascorbic acid intraperitoneally to mice with drug-induced amnesia via the administration of diazepam and scopolamine and to mice that acquired amnesia naturally with age (Parle and Dhingra, 2003). Using the elevated plus maze and the passive avoidance test, the authors concluded that ascorbic acid improved learning and memory in old mice and protected the mice in the group that received the drugs (Parle and Dhingra, 2003). Similarly, other studies have shown that the combination of vitamin C and vitamin E can have beneficial effects preventing memory alterations (Delwing et al., 2006; Hasanein and Shahidi, 2010). However, it has not been possible to demonstrate the reproducibility of these results nor their efficacy in human studies focused on the prevention and treatment of dementia and Alzheimer's disease (Boothby and Doering, 2005; Fillenbaum et al., 2005).

Studies conducted in our laboratory have demonstrated that vitamin C effects on learning and memory are dependent on the redox balance state. When we gave a low dose of vitamin C (50 mg/kg) to healthy rats, their retention latency in the passive avoidance test decreased. Then, when we exposed a group of rats to an acute dose of ozone (0.7 ppm) without vitamin C, the retention latency in the passive avoidance test also decreased. Nevertheless, when we gave the same dose of vitamin C to rats exposed to ozone, the retention latency was similar to that of the control, demonstrating a protective effect of the vitamin (Graphic 1). Subsequently, we compared these results with the lipid peroxidation levels in the hippocampus and we observed a relationship between the oxidative damage and the deficit in the passive avoidance test (Graphic 2). This showed a pro-oxidant effect of low dose vitamin C in a redox equilibrium and an antioxidant effect at any doses in an oxidative stress state (Dorado-Marínez et al., 1998).

**Graphic 1:** **Effects of different doses of vitamin C on memory in redox balance and in oxidative stress**. The retention latency was significantly decreased in the short term memory (STM) and in the long term memory (LTM) in the group that receive 0.7 ppm of ozone (O3) and in the group that receive 50 mg/kg of vitamin C (C50). Meanwhile, at any other doses greater than 50 mg/kg the retention latency were similar to the one of the control group. When any doses of vitamin C were added to the group exposed to ozone, the retention latency in STM and LTM was similar to that of the control group.

**Graphic 2:** **Effects of different doses of vitamin C on lipid peroxidation levels in hippocampus in redox balance and in oxidative stress**. The lipid peroxidation levels mainly increased in the group exposed to ozone (O3) and in the group that receive 50 mg/kg of vitamin C (C50). At any doses of vitamin C greater than 50 mg/kg the effect on lipid peroxidation levels was not as evident as in the C50 and O3 groups. In the groups that receive vitamin C and were exposed to ozone, vitamin C exerted an antioxidant effect (O3 + C50 and O3 + C100), except in the O3 + C200 group.

### Vitamin C and CNS structure

Ascorbate has an important role in the synthesis of collagen and elastin, components of the blood vessels that supply the neural tissue and the basal lamina (Harrison and May, 2009); moreover, the role of ascorbate as an inductor of myelination mediated by Schwann cells has also been demonstrated. Fernandez-Valle et al. observed that adding ascorbate to cultures of Schwann cells with ganglion neurons favored the production of the basal lamina, essential for the induction of myelination, and seemed to induce protein zero mRNA (PZM), which is a major component of myelin; however, the mRNA expression of this protein was not exclusive of the ascorbate culture (Fernández-Valle et al., 1993). It has also been shown that myelination occurs in the presence or absence of ascorbic acid and that the differences under these culture conditions were dependent on laminin (Podratz et al., 2001). Other authors have described that p38, a member of the family of MAP kinases, plays an important role during the early stages of myelination induced by both ascorbate and laminin (Fragoso et al., 2003). Therefore, the main effect of ascorbate on myelination is probably due to the maintenance of the structural integrity of the basal lamina.

### Antioxidant role of vitamin C in CNS

The brain consumes 20% of the total body oxygen and has a high metabolic rate, making it a readily oxidizable tissue (Erecińska and Silver, 2001). These conditions justify the importance of the presence of antioxidants in the brain, which are needed to maintain the redox balance. The distribution of these antioxidants is not uniform since neurons can reach intracellular ascorbate concentrations of 10 mM and a glutathione concentration of 2.5 mM as opposed to what happens in glia where the concentration of ascorbate is 2.5 mM and the one of glutathione is 3.8 mM (Rice and Russo-Mena, 1997). The uneven distribution of ascorbate is due to the fact that SVCT2 is preferentially expressed in neurons; while in astrocytes ascorbate concentrates through the intracellular reduction of DHA which enters the cell via GLUT1. The physiological significance of this unequal distribution is the supply of ascorbate to the neuron. An increase in the expression of mRNA related to the translation of SVCT2 in both neurons and astrocytes has been proven in rats with induced cerebral ischemia, probably as a cellular protective mechanism against oxidative stress induced by ischemia (Berger et al., 2003). Some researchers have studied the interaction of ascorbate with other antioxidants such as α-tocopherol (Niki et al., 1995) and gluthation (Puskas et al., 2000) as well as the possible therapeutic applications of this interaction, e.g., in the prevention of Alzheimer's disease (Morris et al., 1998).

## Role in redox balance

There is a constant balance between oxidants and antioxidants in the body that helps to maintain “redox homeostasis.” This means that when there is an increase the production of ROS, the body's response will be to increase of the activity of endogenous antioxidant systems through a mechanism of redox signaling (Valko et al., 2007). In addition, antioxidants can be obtained from exogenous sources; along with the endogenous antioxidant system, these exogenous antioxidants play an important role in maintaining the redox balance. The endogenous antioxidant systems comprise antioxidant enzymes (e.g., catalase, superoxide dismutase, and glutathione peroxidase) and antioxidant molecules (e.g., glutathione and thioredoxin; Dröge, 2002). Vitamin C, vitamin E and flavonoids are among the exogenous antioxidant molecules ingested in the diet. There are also molecules that function as metal chelators (e.g., lactoferrin and transferrin), avoiding the production of the hydroxyl radical through the Fenton and Haber-Weiss reaction (Valko et al., 2007). An increase in reactive oxygen and nitrogen species that exceeds the ability of the antioxidant system to counteract the increase of ROS leads to an “oxidative stress state.”

The antioxidant effect of ascorbate is due to its ability to donate electrons from both the second and third carbon (Padayatty et al., 2003; Mahfouz and Kummerow, 2004). It has also been demonstrated that ascorbate is more effective than thiols, α-tocopherol, and urate to prevent lipid peroxidation in plasma. Research reported that the higher the concentration of ascorbate in blood is, the greater the time it is required to initiate lipid peroxidation with no pro-oxidant effects, even in ascorbate serum concentrations of 5 mM achievable only parenterally (Frei et al., 1989).

### Recycling mechanisms

To prevent the loss of intracellular concentrations of ascorbate and other antioxidant molecules such as glutathione, cells have recycling mechanisms formed by exogenous antioxidants and the endogenous antioxidant system.

The ascorbyl radical is a relatively stable molecule with an average life of 10–5 s (Buettner, 1993; Padayatty et al., 2003). Its low reactivity is due to the ability of the unpaired electron to resonate between carbons 1′ and 3′ (May, 1999) without interacting with O2 (Bielski and Richter, 1975). Two ascorbyl radicals can react with each other through a dismutation reaction in which one molecule is reduced to ascorbate and the other is oxidized to DHA. Another mechanism involved in the reduction of the ascorbyl radical is the NADH-dependent system mediated by the ascorbyl free radical reductase (AFR reductase) located in the cell membrane (May et al., 2001). Two types of AFR reductases have been described, those which are transmembrane and those found in the inner membrane. Both enzymes seem to be at a convenient location since the ascorbyl radical is formed in the plasma membrane by the reduction of α-tocopherol; thereby counteracting the radicals generated in the intracellular side (May et al., 2001). The α-tocopherol is a lipid antioxidant located near the surface of membranes and lipoproteins where it interacts with ascorbate, which is in the liquid phase of the interface (Niki et al., 1995). By donating an electron, α-tocopherol is oxidized and converted into α-tocopheryl radical, returned to its reduced form by the oxidation of ascorbate interface (Niki et al., 1995).

Thioredoxins are cellular proteins that catalyze the reduction of disulphides in different enzymes (e.g., ribonucleotide reductase) through the transfer of an electron from their thiol group (Arnér and Holmgren, 2000). Thioredoxin reductase is the enzyme responsible for keeping thioredoxin in its reduced form; however, there are reports of the ability of this enzyme to recycle DHA and ascorbyl radical into ascorbate by an NADPH-dependent process in cytosol (Mustacich and Powis, 2000). The glutathione and dihydrolipoic acid are capable of reducing DHA to ascorbate, besides dihydrolipoic acid can also reduce the ascorbyl radical (Kagan et al., 1992; Valko et al., 2007). The relevance of studying these recycling mechanisms is that many of them can be altered in a chronic oxidative stress state, making it more difficult to maintain normal ascorbate concentrations; thereby increasing the requirements for vitamin C in some subjects.

### Pro-oxidant effect of vitamin C

The pro-oxidant ability of ascorbate is associated with the presence of free dissolved metals. A prooxidant effect of ascorbate dependent on the time at which it was administered to rats has been demonstrated (Kang et al., 1998). After injecting paraquat-dichloride intraperitoneally, the researchers recorded an increase in ethane exhalation (oxidative stress marker) and observed lung tissue damage under the microscope. When 10 mg/kg of ascorbate were administered intravenously prior to the injection of paraquat dichloride, a protective effect was observed; however, when ascorbate was administered 1 h after the paraquat dichloride injection, both ethane and tissue damage had increased. The explanation proposed by that study was that the interaction of ascorbate with free metals caused the tissue damage (Kang et al., 1998).

Another study reported an increase in 8-oxoadenine levels (DNA oxidative damage marker) and, paradoxically, a decrease in 8-oxoguanosine levels from basal measurements when supplementing 30 healthy volunteers with 500 mg/day of vitamin C for 6 weeks, compared to the results observed with the placebo group (Podmore et al., 1998). When working with six healthy volunteers, other authors found that the intravenous administration of 750 or 7500 mg of vitamin C did not increase the levels of lipid peroxides nor 8-oxoguanosine (Mühlhöfer et al., 2004). Therefore, some have criticized the results published by Podmore et al. suggesting possible methodological errors (Levine et al., 1998).

Chen et al. demonstrated a susceptibility effect of different types of cancer cells at pharmacological doses (0.3–20 mM) of vitamin C *in vitro*. The mechanism was attributed to the ability of ascorbate to produce H_2_O_2_ in the extracellular space only when the ascorbyl radical levels were >100 nM (Chen et al., 2007). They also found that the production of H_2_O_2_ depended on the presence of redox-active metal centers of proteins (Chen et al., 2005, 2008), which led them to study this effect in a mouse model. They demonstrated a significant decrease in tumor cell growth and tumor weight due to a pro-drug effect of vitamin C (Chen et al., 2008).

A process of ascorbate autoxidation has been proposed when ascorbate is found in its dianionic form. In their review, Du, Cullen and Buettner described that the concentration of dianionic ascorbate increases by a factor of 10 for every pH unit increase (Du et al., 2012). An increased susceptibility to auto-oxidation of dianionic ascorbate has been shown as well (Williams and Yandell, 1982); however, this process does not occur under physiological pH (Buettner, 1988). The possible effect of dianionic ascorbate under pathological conditions with altered pH is yet to be determined.

## Clinical perspective

Given the effect of vitamin C on normal physiology, it is apparent that it plays a role in the maintenance of homeostasis. Nevertheless, it has not been possible to unify the criteria for its clinical use as previous studies have not taken into account the variability of its antioxidant effect, which depends on the redox state of the patient, the dose, and the right route of administration to achieve pharmacological concentrations.

We consider it necessary to continue the study of the therapeutic effects of vitamin C on neurodegenerative diseases, chronic inflammatory diseases, and cancer using vitamin C as a support for patients to decrease the oxidative stress caused by pathological entities.

## Conclusions

The pharmacokinetic properties of ascorbate are intimately related with the functions it performs in tissues since its distribution and concentration in the different organs of the body depend on their requirements of vitamin C. In addition, there exists a specific distribution pattern of ascorbate in each organ which, in brain regions as the *substantia nigra*, is yet to be fully explained. This region has the lowest levels of vitamin C in the brain, a major topic due to the relationship that has been established between oxidative stress and Parkinson's disease.

In addition, the distinction between physiological and pharmacological doses of vitamin C, determined by the route of absorption as well as by the pro-oxidant and antioxidant effect of different doses of vitamin C dependent of the redox balance of the individual, allows us to understand why some previous studies have failed to demonstrate the health benefits of vitamin C.

Finally, the role of vitamin C in health is related to the maintenance of the internal microenvironment determined by the redox balance, proven to be altered in diseases such as obesity, cancer, neurodegenerative diseases, hypertension and autoimmune diseases. This role should be the focus of future research using vitamin C as an adjunct in patient treatment.

### Conflict of interest statement

The authors declare that the research was conducted in the absence of any commercial or financial relationships that could be construed as a potential conflict of interest.
